This article has been retracted.

# The effects of sildenafil in maternal and fetal outcomes in pregnancy: A systematic review and meta-analysis

**DOI:** 10.1371/journal.pone.0219732

**Published:** 2019-07-24

**Authors:** Raquel Domingues da Silva Ferreira, Romulo Negrini, Wanderley Marques Bernardo, Ricardo Simões, Sebastião Piato

**Affiliations:** 1 Department of Obstetrics & Gynaecology, Irmandade Santa Casa de Misericórdia de São Paulo, São Paulo, Brazil, São Paulo; 2 Department of Obstetrics & Gynaecology, Hospital Israelita Albert Einstein, São Paulo, Brazil, São Paulo; 3 Medicine Department, Universidade de São Paulo, São Paulo, Brazil, São Paulo; University of Missouri Columbia, UNITED STATES

## Abstract

**Background:**

The number of studies associating the use of sildenafil in gestation is increasing. This drug inhibits phosphodiesterase type 5 (PDE5), an enzyme responsible for degradation of nitric oxide, and its efficacy is greater in the placental territory, as the maternal side of the placenta have more PDE5 than other sites. For this reason, promising results have been observed related to the prevention of preeclampsia and intrauterine growth restriction and to improvement of maternal-fetal morbidity in cases of placental insufficiency.

**Objective:**

To evaluate the benefits of using sildenafil in pregnancy.

**Searched strategy:**

MEDLINE, ClinicalTrials.gov, Embase, LILACS and Cochrane databases were searched through September 2018. There was no restriction in language or year of publication. This study was registered in PROSPERO (CRD42017060288).

**Selection criteria:**

Randomized clinical trials which used sildenafil for treatment or prevention of obstetric diseases compared with placebo were selected.

**Data collection and analysis:**

The results were obtained using the inverse variance method for continuous variables and Man-Whitney for categorical variables.

**Main results:**

Among a population of 598 pregnant women from the seven clinical trials included, 139 had pre-eclampsia, 275 had intrauterine growth restriction, and 184 had oligohydramnios. A significant increase of 222.58 grams [27.75 to 417.41] was observed in the fetal weight at birth of patients taking sildenafil. The other outcomes did not show any statistical significance. This may be due to the small number of patients used in each study and the great heterogeneity between the groups.

**Conclusions:**

Sildenafil could be associated with increasing fetal weight at birth in placental insufficiency despite the limitations of this meta-analysis, even though more studies in this field are needed to introduce this drug into obstetric clinical practice.

## Introduction

Sildenafil has been used for a long time for male erectile disorder. This drug potentiates the action of nitric oxide by promoting the inhibition of phosphodiesterase type 5, leading to a powerful vasodilator effect [1]. Therefore, there are studies involving this drug in various situations, ranging from pulmonary hypertension to the improvement of the performance of athletes at altitude [2,3].

Obstetrics concerns many diseases due to insufficient placental vascularization and using sildenafil in this field could have several benefits [4]. Several animal studies show that sildenafil could affect utero-placental circulation, resulting in improvement in the maternal-fetal exchanges [5,6]. Despite the reduced number of pregnant women taking sildenafil even for maternal cardiac indications, there is no report of teratogenicity or any relevant adverse effect [7–9].

Pre-eclampsia (PE) and fetal growth restriction (FGR) are pathologies in which there are clear blood placental supply difficulties with potentially disastrous consequences to the fetus and the mother [10,11]. As these infants are usually born very preterm, PE and FGR are the major cause of perinatal mortality and morbidity worldwide. We are currently able to predict, with some confidence, the risk of severe PE and FGR based on clinical, ultrasonography and biochemical markers. However, we still do not have an adequately effective form of treatment in all cases [12,13]. The ASPRE trial demonstrated that administration of aspirin resulted in a 62% reduction in the incidence of preterm PE but had no significant effect on the incidence of term PE [14].

The objective of the present study was to verify obstetric uses of sildenafil citrate through a systematic review and meta-analysis, aiming to identify new possibilities of treatment for prevalent obstetric conditions, such as PE and FGR, which are associated with high rates of maternal and fetal morbidity and mortality worldwide.

## Sources

This systematic review and meta-analysis was reported according to PRISMA (Preferred Reporting Items for Systematic Reviews and Meta-Analyses), and it was registered in the international database PROSPERO (International Prospective Register of systematic reviews), registration number: CRD 42017060288 [15,16].

The MEDLINE through PubMed, ClinicalTrials.gov, Embase, LILACS and Cochrane databases were searched. A gray and manual search was also performed via analysis of book chapters, theses, reference references, guidelines and reviews. The last search was performed in September 2018. For the MEDLINE and Embase we used the following terms: “(Pregnancy OR Pregnancies OR Gestation OR Gravidity OR Eclampsia OR Preeclampsia OR Edema Proteinuria Hypertension Gestosis OR EPH Toxemia OR EPH Gestosis) AND (Sildenafil OR Tadalafil)”. For LILACS we used: (Pregnan$ OR Gesta$ OR Gravidity OR Eclampsia OR Preeclampsia OR "Edema Proteinuria HypertensionGestosis" OR "EPH Toxemia" OR "EPH Gestosis" OR gravidez OR embarazo) AND (Sildenafil OR Tadalafil). For the ClinicalTrials.gov and Cochrane databases, the following descriptors were used: “pregnancy AND sildenafil”.

The patients included were pregnant women, with no restriction regarding gestational age. The intervention studied was the use of sildenafil in comparison with placebo. The results sought were maternal and fetal outcomes, such as weight at birth, gestational age at birth, indications for delivery, umbilical artery pulsatility index, neonatal mortality and side effects. Only randomized clinical trials were included with no cut-off date or language restriction.

The selection of manuscripts, as well as the evaluation of titles and abstracts, was conducted by two blinded researchers working independently and strictly observing the inclusion and exclusion criteria. Only articles for which we had access to the full text were included. The bibliographies of the included and excluded studies were evaluated to find potentially relevant studies that had not been identified by the initial search strategy. Data were extracted and compiled into tables for further analysis and description.

The information withdrawn from each trial included the author, year of publication, population studied, intervention and control group, outcomes and follow-up time. The analyzed outcomes were fetal weight at delivery, indication of the resolution of pregnancy, gestational age at birth, umbilical artery pulsatility index, neonatal mortality and medication tolerance (side effects).

The risk of bias for individual studies was determined based on Cochrane Risk of Bias Tool for Randomized Controlled Trials by assessing the following aspects: focal issue, appropriated randomization, concealment allocation, double blind, losses (less than 20%), prognostic or demographic characteristics, intention to treat analysis and sample calculation [17]. The Jadad index was also calculated for each study [18].

The principal summary measures employed were risk differences for categorical variables and median differences for continuous variables. A 95% confidence interval was used. A meta-analysis was performed using Review Manager Software (RevMan) 5.3.

The analysis began with a fixed-effects model, and the Mann-Whitney test and inverse-variance weighting were applied for categorical and continuous variables, respectively. After heterogeneity had been calculated (I^2^), a random-effects model was used if heterogeneity was greater than 50% and if there was no publication bias to be treated and identified by the Egger test through funnel plots [19].

## Results

### Study selection

A total of 524 articles were identified through an initial search in the databases cited above. After excluding duplicate papers, 242 articles remained. In the initial analysis in which titles and summaries were considered, 197 articles were excluded because they were not related to the obstetric use of sildenafil or used it experimentally in animals. The full text of the 45 remaining studies was then analyzed. Based on this assessment, 38 studies were excluded due to the following reasons: 15 were ongoing, eight were specialists’ opinions; five were case reports; four were cohort studies, two were not availble; and four were systematic reviews. Ultimately, seven relevant trials were selected and meta-analyzed, as shown in Fig 1.

**Fig 1:** PRISMA Flowchart of recovery and selection of studies.

The population of the selected trials consisted of 598 pregnant women, all with comorbidities, among them 139 with pre-eclampsia [20,21], 275 with intrauterine growth restriction [21,22–25], and 184 with oligohydramnios [26].

The gestational age of the initial treatment ranged from 24 to 30 weeks. All of the pregnant women used oral sildenafil, with doses ranging from 50 mg to 150 mg daily. With the exception of one study [26], all patients used a pill similar to sildenafil as the placebo. The follow-up time of all the studies was from the day of recruitment until birth, except for one study that did not follow up patients until delivery [22].

The outcomes were fetal weight at birth, gestational age at birth, indications of gestational resolution, umbilical artery pulsatility index, neonatal mortality, and side effect of medication use. Table 1 summarizes the characteristics of the seven selected trials.

**Table 1:** Characteristics of the studies.

Study (year)	Population (n)	Intervention—Sildenafil (n)	Control—Placebo (n)	Analyzed outcomes	Follow up time
Samangaya (2009)^20^	Women with pre-eclampsia and gestational age between 24 and 34 weeks. (39)	Sildenafil 20 to 80 mg oral daily, (19)	Placebo orally. (20)	Fetal weight at birth, indication of pregnancy resolution, umbilical artery PI, neonatal mortality, and side effects.	From recruitment to the day of birth.
Von Dadelszen (2011)^23^	Pregnant women with severe early onset intrauterine growth restriction. (27)	Sildenafil 25 mg every 8 hours orally from recruitment to the day of birth. (10)	Placebo orally. (17)	Gestational age at birth, neonatal mortality, and side effects.	From recruitment to the day of birth.
Dastjerdi (2012)^22^	Pregnant women with intrauterine growth restriction—percentile 3. (59)	Oral sildenafil 50 mg, one single dose. (29)	Placebo orally, one single dose. (30)	Umbilical artery pulsatility index (PI), neonatal mortality and side effects.	No follow up.
Trapani (2016)^21^	Women with pre-eclampsia and single gestation between 24 and 33 weeks of gestation. (100)	Sildenafil 50 mg every 8 hours orally from recruitment to the day of birth. (50)	Placebo orally. (50)	Fetal weight at birth, indication of pregnancy resolution, umbilical artery PI, neonatal mortality, and side effects.	From recruitment to the day of birth.
El Sayed (2017)^24^	Pregnant women with fetal growth restricition due to placental insufficiency with 24 weeks or more. (54)	Oral sildenafil 50 mg, daily. (27)	Placebo orally. (27)	Fetal weight at birth, gestational age at birth, umbilical artery PI, neonatal mortality, and side effects.	From recruitment to the day of birth.
Maher (2017)^26^	Pregnant women with oligohydramnios (ILA <5 cm), older than 30 weeks. (184)	Sildenafil 25 mg orally every 8 hours and intravenous hydration. (89)	Intravenous hydration. (95)	Fetal weight at birth, neonatal mortality, and side effects.	From recruitment to the day of birth.
Sharp (2018)^25^	Pregnant women with fetal growth restriction (percentile <10) and absent or reversed end-diastolic flow in umbilical artery on Doppler, from 22 to 29 weeks and 6 days. (135)	Sildenafil 25 mg every 8 hours orally from recruitment to 32 weeks or birth (70)	Placebo orally. (65)	Fetal weight at birth, gestational age at birth and neonatal mortality.	From recruitment to the day of birth.

^n^Number of patients.

There was no appropriate randomization and blind allocation in approximately one-third of the trials. Losses greater than 20% of the initial sample occurred in two studies [20,22]. Both the demographic characteristics of the sample and the measured outcomes were adequately explained in all of the selected trials. However, only one presented a sample calculation [21], and an analysis by intention to treat was conducted in four trials [21,24–26].

The risk analysis of bias is outlined in Fig 2, which shows separately the risks of each bias between each trial, and in Fig 3, which presents the percentage of each bias among all trials.

**Fig 2:** Risk of bias for each study.

**Fig 3:** Risk of bias for all studies.

### Analysis of outcomes

Fetal birthweight was analyzed in five trials [20,21,24–26], selected for the meta-analysis for a total of 508 patients, with 255 in the sildenafil group and 253 in the placebo group. For the sildenafil group, an increase of 75.55grams [49.27 to 101.83 grams] in fetal weight at birth was observed (Fig 4). However, as a high heterogeneity between the studies was identified (I^2^ = 96%) and the Egger test through the funnel plot (Fig 4) demonstrate that there was not only one trial in which the results differs from the others, the analysis was based on the random model, as shown in Fig 5. This resulted in a significant increase of 222.58 grams [27.75 to 417.41 grams] in fetal weight among women using sildenafil during gestation, with the start use between 20 and 30 weeks, until the delivery (Fig 5).

**Fig 4:** Fetal weight at birth: Analysis by the fixed-effects model and funnel plot. SD: standard deviation; IV: variance inverse; CI: confidence interval.

**Fig 5:** Fetal weight at birth—Analysis by the random-effects model. SD: standard deviation; IV: variance inverse; CI: confidence interval.

Gestational age at birth was assessed by two trials [23,24] among 81 pregnant women, 44 in the placebo group and 37 in the sildenafil group. As high heterogeneity was observed between the studies (I^2^ = 93%), the analysis was based on the random-effects model, as shown in Fig 6. No differences were observed between the two groups in relation to gestational age at birth (-0.12 [-2.84, 2.59]).

**Fig 6:** Gestational age at birth. SD: standard deviation; IV: variance inverse; CI: confidence interval.

Four trials [20–22,24] evaluated the umbilical artery pulsatility index (PI) between sildenafil and placebo groups, totaling 278 patients, with 125 in the former and 153 in the latter. On average, a 12% reduction [7% to 18%] in the umbilical artery PI in the sildenafil group was found (Fig 7). However, there was high heterogeneity among the studies (I^2^ = 91%) and the Egger test revealed an outlier in the funnel plot [24], as shown in Fig 7. Therefore, after excluding the outlier [24] the heterogeneity remained high (I^2^ = 72%), so the study was maintained, and the random model method was used, as shown in Fig 8. There was no difference between the groups regarding the umbilical artery PI (0.04 [-0.18, 0.27]).

**Fig 7:** Umbilical artery pulsatility index—Analysis by the fixed-effects model and funnel plots. SD: standard deviation; IV: variance inverse; CI: confidence interval.

**Fig 8:** Umbilical artery pulsatility index—Analysis by the random-effects model. SD: standard deviation; IV: variance inverse; CI: confidence interval.

Assessment of reasons for parturition among sildenafil and placebo groups was performed in two trials [20,21]. A total of 139 pregnant women, 69 in the sildenafil group and 70 in the placebo group, were analyzed. In the case of indication of delivery due to fetal distress, there was no difference between the groups (-0.03 [-0.17, 0.12]), as shown in Fig 9. Similarly, in relation to the indication of labor due to maternal laboratory abnormality, such as creatinine>2 mg/dl, thrombocytopenia and/or increase in liver enzyme levels, there was no difference between the groups (Fig 10; 0.00[-0.14, 0.15]). An indication of gestational resolution due to imminent eclampsia was also analyzed. As shown in Fig 11, there was no difference between the groups (-0.05 [-0.20, 0.10]).

**Fig 9:** Indication of delivery due to fetal distress. SD: standard deviation; M-H: *Mann-Whitney*; CI: confidence interval.

**Fig 10:** Indication of labor due to maternal laboratory test abnormality. SD: standard deviation; M-H: *Mann-Whitney*; CI: confidence interval.

**Fig 11:** Indication of delivery due to imminent eclampsia. SD: standard deviation; M-H: *Mann-Whitney*; CI: confidence interval.

The number of neonatal deaths was evaluated in all of the selected trials [20–26], with a total of 598 pregnant women, 294 in the sildenafil group and 304 in the placebo group. However, no significant difference was observed between the groups, as shown in Fig 12 [-0.01 (-0.05, 0.03)].

**Fig 12:** Neonatal mortality. SD: standard deviation; M-H: *Mann-Whitney*; CI: confidence interval.

Headache as a side effect of the use of the prescribed medication was reported in six clinical trials [20–24,26], totaling 463 patients, 224 and 239 in the sildenafil and placebo groups, respectively. Although no difference between the groups in the occurrence of headache was found (0.04 [-0.02, 0.09]; Fig 13), heterogeneity between the groups was high (I^2^ = 69%). An outlier [26] was identified based on the Egger test, through the funnel plot, as shown in Fig 13. Removing the outlier [26] from the meta-analysis resulted in a significant decrease in heterogeneity (I^2^ = 7%), evidencing publication bias for the article in question. However, as shown in Fig 14, the result remained the same, with no difference between the groups (0.06 [-0.03, 0.15]).

**Fig 13:** Headache as a side effect—Analysis by the fixed-effects model and funnel plots. SD: standard deviation; M-H: *Mann-Whitney*; CI: confidence interval.

**Fig 14:** Headache as a side effect—Analysis after removing the outlier. SD: standard deviation; M-H: *Mann-Whitney*; CI: confidence interval.

## Discussion

The use of sildenafil for several purposes has occurred for many years and there are some suggestions concerning its benefits in obstetric pathologies, especially with regard to the vasodilating effect of this medication. Therefore, the present research aimed to identify the real benefits attributed to this drug in the pregnancy-puerperal cycle by the most reliable scientific methodology known, which is the systematic review with meta-analysis.

During this search, we found four systematic reviews published. As most the clinical trials related to this subject were done recently in the last two years, all these reviews included experimental studies and case reports. Besides that, only the last review published did a meta-analysis of the results, which showed that sildenafil has the potential to improve fetal growth during suboptimal intrauterine growth conditions [27]. The maternal tolerance was analyzed by Dunn et al, and its results are similar to ours, considering that there was no severe adverse maternal side effects by the use of sildenafil in pregnancy and the available evidence suggests that it is a safe medication supported by its potential as therapy for selected maternal and fetal disorders [28].

Although there are many experimental animal studies, as well as in vitro studies using sildenafil in pregnancy, they were excluded to afford more credibility to this meta-analysis, which makes this an original work. Unfortunately, there are few randomized clinical trials concluded until now and all of them had limited samples. The largest one had only 184 patients.

Despite the fetal weight was described in six of the seven selected trials, only in four of them it was analyzed and in only two it had a statistically significant result [24,26]. Sildenafil was associated with a significant increase in abdominal circumference growth velocity in von Dadelzen et al trial [23], but the weight at birth was not mentioned. Fetal weight at birth was a secondary endpoint in Samangaya et al trial [20] and it probably did not show a statistically significant result because of heterogeneity of the recruited population and the limited time of the use of the drug, considering that 66% of the deliveries were precipitated. The trial of Trapani et al [21] did not demonstrate significance between sildenafil and placebo groups in fetal outcomes and this was considered to be the result of a lack power given the small number of cases and the late start of medication. Sharp et al [25] recruited a severe fetal growth restriction population, with umbilical Doppler artery abnormalities, and it was given a low dose of sildenafil, as discussed in by Walton et al in their experimental study [29]. Maybe therapeutic dose of was not achieved and these could have contributed for the non-significant results.

Although all studies in this meta-analysis included pregnancy disorders that arise in a background of uteroplacental insufficiency, they all have a variety of manifestations and probably different pathophysiologies, which weakens the results. The conclusions were limited by the lack of studies in this field, which made a separately analysis by each disease infeasible.

Even with all these risk bias involved, the main benefit of sildenafil to pregnant women reported in this meta-analysis is an increase in fetal weight at birth; thus, an indication for the use of this drug might be pregnancies with fetal growth restriction (FGR). This is remarkable, as it is well known that smaller fetuses present the largest rates of complications in both the short and long term [30]. For example, newborns with weights below the 10^th^ percentile between 32 and 42 weeks of pregnancy are three to six times more likely to have cerebral palsy than those weighing within the 25^th^ and 75^th^ percentiles [31]. Furthermore, low birth weight results in chronic diseases, especially cardiovascular disease [32].

Once FGR is established and diagnosed, sildenafil may be able to reduce fetal effects. However, more important is the possibility of the drug preventing low birth weight in women at high risk for developing FGR. This potential may be forthcoming, considering that it is possible to determine the probability of developing FGR based on the levels of angiogenic factors in maternal blood [33]. We are still waiting the final results of the STRIDER multicenter trials that are researching sildenafil therapy for early-onset intrauterine growth restriction pregnancies [34]. The scientific community was alerted with recent news concerning the death of eleven newborns from women who were given sildenafil in the Dutch trial [35]. The case remains uncertain and the trial was suspended at the moment. One of the questions to be raised is the patient’s selection criteria, which was pregnant women with a severe early onset fetal growth restriction. This population has itself a higher risk of death considering it’s morbidities. This is also an important warning to the community that this medication is not yet approved for use in obstetrical clinical practice for the purpose of treating or preventing placental insufficiency (either fetal growth restriction or preeclampsia) and therefore should not be done outside the scope of clinical trials.

The great unknown that still persists is related to the ideal timing of using sildenafil. Whether the use should be instituted when the preeclampsia or fetal growth restriction is observed or if the treatment should be done preventively during the placentation, as proposes Larré et al [36]. The second option seems more plausible pathophysiologically. Therefore, it is necessary to identify the risk group for preeclampsia and/or fetal growth restriction, a condition that is fortunately possible, based on the levels of angiogenic factors in maternal blood and uterine Doppler flow [37]. Besides that, Brownfoot et al reported that sildenafil is associated with a reduction in circulating sFlt-1 levels in a patient with preterm preeclampsia [38].

However, none of the studies included in this meta-analisys introduced sildenafil in the first trimester of pregnancy, during the placentation. Furthermore, in the most of them the fetal weight was more than 1000g, when perinatal outcomes are usually good. It could bring the possibility that perhaps response to sildenafil may be related to a less severe pathology.

In addition to the increase in fetal weight at birth, other outcomes, including gestational age at birth, umbilical artery pulsatility index, indication of the resolution of gestation, neonatal mortality and side effects, can be considered secondary. Despite a lack of significant results, all studies reported a beneficial tendency in the sildenafil group. In addition, the small sample sizes, as well as the high heterogeneity present, a revealed by the meta-analysis, may have contributed to the low level of statistically relevant data.

In this sense and considering the limits of this systematic review, even though we followed exactly the PRISMA recommendations, tried to use the most variety of keywords possible and committed to be as impartial as possible we know that it is possible that some articles may have been lost in these search, which could compromise our results. Furthermore, it was observed that some studies did not present all the analytical data available, and each had a different method of measuring certain outcomes, which rendered the comparison a difficult and challenging task. Moreover, there were significant differences in the methodologies used. The patients recruited ranged from those in early pregnancy to after 30 weeks of gestation, and this was likely the reason why one of the articles (Maher et al) increased the heterogeneity and was excluded from some analyses. Furthermore, the patients had different obstetric diseases, including fetal growth restriction, pre-eclampsia and oligohydramnios, all of which lead to placental insufficiency. Despite all these limitations and bias risks, the meta-analysis showed that fetal weight at birth increased by using sildenafil in cases of placental insufficiency.

It should also be noted that no studies involved long-term follow-up of newborns, which prevented us from concluding whether there were any repercussions of the drug in childhood. However, considering the security of the use of this medication in pregnancy and given that no teratogenic effect has been verified, sildenafil might constitute a new treatment for many serious obstetric diseases, particularly preeclampsia and FGR.

Despite these results, further clinical trials adequately randomized with similar methodologies and including the same pregnancy disorders are still necessary to evidence the increasing in fetal weight at birth in cases of placental insufficiency. Besides that, we await the results the STRIDER multicenter trials to clarify if there is benefits in using Sildenafil for early-onset intrauterine growth restriction pregnancies.

## Conclusion

This meta-analysis evidenced that sildenafil could be associated with increasing in fetal weight at birth despite the few number of studies and the variety population included without considering the diversity etiologies for placental insufficiency, such as fetal growth restriction and preeclampsia. More studies in this field are needed to introduce this drug into obstetric clinical practice, especially after the Dutch trial incident.

## Supporting information

S1 File Prisma Checklist. SD: standard deviation; IV: variance inverse; CI: confidence interval; M-H: *Mann-Whitney*.
(PDF)
